This article has been retracted.

# MicroRNA-505-5p functions as a tumor suppressor by targeting cyclin-dependent kinase 5 in cervical cancer

**DOI:** 10.1042/BSR20191221

**Published:** 2019-07-26

**Authors:** Elena Kapora, Shujun Feng, Wei Liu, Indira Sakhautdinova, Bo Gao, Wenhua Tan

**Affiliations:** 1 Department of Gynecology and Obstetrics, The Second Affiliated Hospital of Harbin Medical University, Harbin, Heilongjiang 150086, China; 2 First department of Gynecology and Obstetrics, Bashkir State Medical University, Ufa, Republic of Bashkortostan 450008, Russia

**Keywords:** Cervical cancer, cell invasion, cell migration, cell proliferation, CDK5, miR-505-5p

## Abstract

MicroRNAs (miRs) are considered to be tumor suppressors or oncogenes as they regulate cell proliferation, migration, invasion, and differentiation. Recently, microRNA-505 (miR-505) has been reported as being involved in the progression of several human cancers. In the present study, we aim to investigate the expression rate and functional role of miR-505-5p in cervical cancer (CC) to determine its significance regarding the disease’s development.

The expression of miR-505-5p and cyclin-dependent kinase 5 (CDK5) in specimens of patients with CC and CC cell lines was examined by quantitative real-time PCR (qRT-PCR) and Western Blot. The relationship between miR-505-5p and CDK5 was verified by luciferase reporter assay. Cell counting kit-8 (CCK-8) assay, Scratch wound healing assay and transwell assay were used to detect the roles of miR-505-5p and CDK5 in CC cell functions. Western Blot was utilized to explore the epithelial–mesenchymal transition (EMT) markers.

The result showed that in CC tissues and CC cell lines miR-505-5p was down-regulated while CDK5 level was up-regulated. MiR-505-5p was closely correlated with the metastasis-associated clinicopathological features. Overexpression of miR-505-5p inhibited cell viability, cell metastasis and EMT in CC cells. CDK5 was confirmed as a direct target of miR-505-5p and inverse relationship between them was also observed. Overexpression of CDK5 reduces the inhibitory effects of miR-505-5p in CC.

Taken together, these results determine that miR-505-5p is a tumor suppressor miRNA which regulates tumor cell proliferation, migration, and invasion via binding to the functional target CDK5 and demonstrates its potential for future use in the treatment of CC.

## Introduction

According to statistics generated by the American Cancer Society in 2015, the fatality rate of cervical cancer (CC) is the second highest among female patients [1]. CC is also ranked 9th of all cancers in terms of mortality, and accounts for 266,000 deaths/year worldwide. According to estimates, the highest new CC incidence rate in 2012 was in South-Central Asia (151.8/100,000), which had the world’s highest estimated number of cancer deaths of 82.2/100,000 [2]. The World Health Organization recognizes three categories of epithelial cervical tumors: squamous cell carcinoma, accounting for 70–80% of CCs; adenocarcinoma, accounting for 20–25% of CCs; and other tumors (adenosquamous carcinoma, neuroendocrine tumors, and undifferentiated carcinoma). Despite considerable advances in treatment, the 5‐year survival rate for cervix uteri cancers varies, from below 40% to more than 70% across different countries [3–5]. Therefore, it is essential to investigate the mechanisms involved, and to identify new molecular markers for personalized treatment leading to advances in CC therapy.

MicroRNAs (miRNAs) are short endogenous non-coding molecules with a length of around 19–23 nucleotides. They regulate gene expression by binding to complementary sequences in the untranslated regions (UTRs) of target mRNAs [6]. Today, it is known that miRNAs can be involved in carcinogenesis, either as oncogenes or as suppressors [7].

There is increasing evidence supporting the view that miRNAs are frequently dysregulated in CC, that they act as critical regulators of carcinogenesis and cancer progression, and that they are useful as diagnostic and prognostic markers for CC [8,9]. However, our understanding of how miRNAs regulate CC development and progression – particularly how they affect CC metastasis – remains limited. Recent studies demonstrate that microRNA-505 (miR-505) is dysregulated in different types of human cancers, including breast cancer, colorectal cancer, prostate cancer, endometrial cancer, bladder cancer, and hepatocellular carcinoma, among others [10–22]. Furthermore, miR-505 expression levels in plasma [21] and in whole blood [22] could be used as a potential non-invasive biomarker for bladder and pancreatic cancer. Previous reports show that miR-505 expression decreases in CC tissues, and that overexpression leads to inhibition of tumor growth and invasion by targeting FZD4 [23]. Despite these findings, the role played by miR-505-5p in CC progression and epithelial–mesenchymal transition (EMT) process remains elusive.

## Materials and methods

### Human tissues

CC tissues and normal cervical tissues were obtained from patients who underwent surgery between December 2015 and July 2017 at the Second Gynecology Department, Second Affiliated Hospital of Harbin Medical University (Heilongjiang Province, China). Patients diagnosed with CC (*n*= 60) and with other non-cancerous gynecological diseases (*n*=60) at the Second Affiliated Hospital of Harbin Medical University were included in the present study. Only those specimens taken from patients with newly diagnosed CC, who had not received prior treatment, were included in the study. After resection, all 120 tissue samples were immediately frozen in liquid nitrogen and stored at −80°C until RNA extraction. Clinical and pathological data, including age, FIGO (International Federation of Gynecology and Obstetrics) stage, tumor size, lymph node status, and histology grade, were retrieved from the patients’ records.

### Cell culture and transfection

Five human CC cell lines, epidermoid cervical carcinoma (Ca-Ski), adenocarcinoma (HeLa), squamous cervical carcinoma (SiHa, C-33A), cervical carcinoma (HT-3), and normal human cervical cell line (Ect1/E6E7), were obtained from the Chinese Academy of Sciences’ Cellbank (Shanghai, China). Cells were cultured in Dulbecco’s modified Eagle’s medium (HyClone; GE Healthcare Life Sciences, Logan, UT, U.S.A.). The culture media were supplemented with 5% (vol/vol) fetal bovine serum (FBS) and 1% penicillin/streptomycin. The cell lines were then incubated at 37°C in a humidified atmosphere containing 5% CO2. All experiments used cells with a passage number <20.

Cells were each transfected with miR-505-5p mimics and negative control miRNA (NC), obtained from Shanghai GenePharma Co., Ltd., (Shanghai, China) using Lipofectamine2000 and Opti-MEM (Invitrogen, Carlsbad, U.S.A.), according to the manufacturer’s protocol. The miR-505-5p mimics sequence: sense 5′-GGGAGCCAGGAAGUAUUGAUGU-3′, antisense 5′-AUCAAUACUUCCUGGCUCCCUU-3′; negative control had the following sequence: sense 5′-UUCUCCGAACGUGUCACGUTT-3′, antisense 5′-ACGUGACACGUUCGGAGAATT-3′. For the cyclin-dependent kinase 5 (CDK5) experiments, CDK5 overexpression sequence was inserted into pcDNA 3.1 vector. The transfection sequence was synthesized by Cyagen (Beijing, China).

### RNA extraction and quantitative real-time PCR

Total RNA was isolated from cultured cells and tissues using Trizol reagent (Invitrogen; Thermo Fisher Scientific, Inc., Waltham, MA, U.S.A.) according to the manufacturer’s instructions. RNA concentration and purity were determined using a NanoDrop spectrophotometer (Thermo Fisher Scientific, Inc.). Total RNA was then reverse transcribed into cDNA using a cDNA reverse transcription kit (TOYOBO Bio-Technology, Co., Ltd., China), according to the manufacturer’s protocol.

Quantitative real-time PCR (qRT-PCR) was performed on a 7500 Fast Real-Time PCR System (Applied biosystems) using the SYBR PrimeScript RT-PCR kit (TOYOBO Bio-Technology, Co., Ltd., China) with specific primers. Small nuclear RNA (snRNA) U6 or GAPDH was used as an internal control. The primers used for qRT-PCR were as follows: miR-505-5p, forward primer: 5′-GTA ATC GGG AGC CAG GAA GT-3′, and reverse primer: 5′-GTG TCG TGG AGT CGG CAAT-3′; U6 forward primer: 5′-ATTGGAACGATACAGAGAAGATT-3′; and reverse primer: 5′-AGGAACGCTTCA CGAATTTG -3′; CDK5 forward primer: 5′- ATTAGCAGGTTCTGGGGCTT -3′, and reverse primer: 5′-AATGGTGACCTCGATCCTGA 3′; GAPDH forward primer: 5′-GGAG CGA GAT CCCTCCAAAAT-3′, and reverse primer: 5′-GGCTGTTGTCATACTTCTCATGG-3′. Sybergreen master mix was used as a detection dye. PCR conditions are as follows: holding stage incubation at 50°C for 2 min, 95°C for 10 min, two-step amplification at 95°C for 15 s, and 60°C for 1 min with 40 cycles; the melting conditions were 95°C for 15 s, 60°C for 1 min, 95°C for 30 s continuous, and cooling at 60°C for 15 s. Amplification of all miRNAs in the samples was carried out according to the manufacturer’s instructions, and analyzed using the Real-Time Light Cycler 7500 software. Each experiment was performed in triplicate. Relative expression fold changes were calculated using the 2^−ΔΔ*C*^_t_ method and normalized to U6 and GAPDH expression.

### Cell migration assay

HeLa and SiHa cells were seeded in 12-well plates and transfected with miR-505-5p mimics and negative control, according to the manufacturer’s instructions. Some cells were co-transfected with pcDNA 3.1-CDK5 and miR-505-5p mimics, either independently or together. Additionally, co-transfection of pcDNA 3.1 empty vector, together with NC, was used as a control.

After 48 h of incubation, cells were seeded for migration assay. A sterile pipette tip was used to scratch the confluent cell layer, thereby creating a linear wound. After cells had been washed three times using phosphate-buffered saline (PBS), and the medium had been changed to FBS free DMEM, cells were further incubated at 37°C. Photos were captured on a light microscope at 40× magnification, 0 and 48 h after wounding.

### Cell invasion assay

The invasive properties of CC cells were measured using a 24-well transwell invasion assay. 24 h after transfection, 1 × 10^5^ cells were resuspended in 140 μl serum-free culture medium and seeded in the top chamber of a transwell (Corning Inc., Corning, NY, U.S.A.) that had been coated with Matrigel (BD Biosciences, San Jose, CA). The bottom chamber was supplemented with a complete medium with 10% FBS. After 48 h of incubation, cells migrated to the other side of the transwell were fixed and stained with hematoxylin and eosin. Invading cells in the lower chambers were photographed at 100× magnification and counted for each well.

### Cell proliferation assay

Cell counting kit-8 (CCK-8) (Dojindo Laboratories, Kumamoto, Japan) was used to detect cell proliferation. Control and cells transfected with desired vectors were seeded into 96-well plates at a density of 1 × 10^3^ cells/well. At desired time points, CCK-8 solution (10 μl) was added to each well and incubated for 2 h at 37°C. Optical density (OD) values were determined using a microplate reader (SM600 Labsystem, Shanghai, China) at 490 nm.

### Luciferase reporter assay

A luciferase assay was carried out to confirm the interaction between miR-505-5p and CDK5. Human HeLa and SiHa cells were seeded into 24-well plates and co-transfected with miR-505 mimics or negative control; they were then cross-transfected with the wild-type CDK5 (CDK5-WT) or mutant sequence (CDK5-MUT) for 48 h. Subsequently, relative luciferase activity was measured using a luciferase reporter assay (Promega, Wisconsin, U.S.A.) according to the manufacturer’s protocol. Results were normalized with Renilla luciferase.

### Western blot

28 h post-transfection, cells were washed twice with cold PBS and lysed with radioimmunoprecipitation assay buffer (RIPA) (Thermo Fisher Scientific, Waltham, MA, U.S.A.) at 4°C for 5 min for further protein extraction. Collected lysates were cleared by centrifugation, and total protein concentration was quantified using the BCA Protein Assay Reagent Kit (Beyotime, Shanghai, China). Equal amounts of protein (80 μg) for each sample were loaded and separated on a 10% sodium dodecylsulphate polyacrylamide gel (SDS/PAGE) before being transferred onto a polyvinylidene difluoride (PVDF) membrane. The membranes were blocked in 5% skim milk and incubated at room temperature for 1 h. The following appropriate primary antibodies – including, anti-Vimentin (ab92547), anti-N-cadherin (ab98952), anti-E-cadherin (ab40772), and anti-CDK5 (ab220214) – were obtained from Abcam (Cambridge, MA, U.S.A.), and anti-β-actin (TA-09) was obtained from ZSGB-BIO (ZSGB Biotechnology, Beijing, China). All primary antibodies were diluted 1:1000 and added to the membranes for overnight incubation at 4˚C. Subsequently, membranes were washed in TBST solution four times before being incubated with horseradish peroxidase (HRP)-conjugated secondary antibodies for 1 h at room temperature. Blots were visualized using the Odyssey CLx Infrared Imaging system (Li-COR Biosciences) and the Image Studio software.

### Statistical analysis

All experiments were performed in triplicate, and the averaged data were presented as mean ± standard deviation (S.D.). The Student’s *t*-test was used to analyze differences between two groups, and two-way ANOVA was used when more than two groups were compared. The correlations between miR-505 and CDK5 expression were analyzed using the Pearson correlation test. Statistical analysis was carried out using a SPSS 22.0 software. *P*-values were calculated, and *P*<0.05 was considered to be statistically significant by two-tailed unpaired student’s *t*-test.

## Results

### MiR-505-5p is down-regulated in human CC tissue samples and correlates with poor prognosis in patients with cervical cancer

QRT-PCR was performed to measure miR-505-5p expression levels in 60 CC samples and 60 histologically normal cervical tissues. Results showed that miR-505-5p in human CC tissues was significantly lower than in healthy controls (*P*<0.01; Figure 1A).

**Figure 1:** MiR-505-5p expression is down-regulated in cervical cancer **(A)** Cervical tissues extracted from human patients. QRT-PCR was used to compare miR-505-5p expression levels between CC tissues (Cervical cancer, *n*=60) and non-cancerous cervical tissues (Normal cervical, *n*=60) (^**^P<0.01; by Student’s *t*-test vs normal cervical tissues). **(B)** QRT-PCR was applied to measure miR-505-5p expression levels in *in vitro* cervical cancer cell lines, Ca-Ski, HeLa, SiHa, C-33A and HT-3, and then normalize them to miR-505-5p expression in a non-carcinoma cervical epithelial cell line, Ect1/E6E7 (^*^P<0.05, **P<0.01; by Student’s *t*-test vs Ect1/E6E7).

To investigate the clinical value of miR-505-5p, and to find its prognostic significance in CC, we collected the clinical characteristics of patients diagnosed with CC at the Second Affiliated Hospital of Harbin Medical University. Based on the expression levels of miR-505-5p in CC, patients were divided into low (*n*=30) and high (*n*=30) miR-505-5p expression groups. The median value was used to divide the patients into two equally sized groups with low (below median) and high (above median) levels of miR-505-5p expression.

Our findings showed associations between miR-505-5p expression with FIGO stage (*P*=0.016), tumor size (*P*=0.034), lymph node metastasis (*P*=0.019), and histology grade (*P*=0.020) in patients with CC (Table 1). These results suggest that down-regulation of miR-505-5p might be used as a novel marker for CC prognosis and progression.

**Table 1:** Associations of miR-505-5p expression with the clinicopathological features of patients with cervical cancer

Characteristics	miR-505-5p			
	No. of cases	Low level	High level	*P*-value
Age (years)				0.787
<50	39	19	20	
≥50	21	11	10	
FIGO				0.016
I–II	38	14	24	
III–IV	22	16	6	
Tumor size (cm)				0.034
<4	37	14	23	
≥4	23	16	7	
Involved lymph node				0.019
Negative	26	8	18	
Positive	34	22	12	
Histology grade				0.020
Well and moderate	32	11	21	
Poor	28	19	9	

### Expression level of miR-505-5p in CC cell lines

To examine whether miR-505 is down-regulated in CC cell lines, we first determined its expression level in *in vitro* cervical cancer cell lines: Ca-Ski, HeLa, SiHa, C-33A, and HT-3 cells using qRT-PCR assays. The expression levels of miR-505 were measured and compared with the expression level in a non-carcinoma cervical epithelial cell line, Ect1/E6E7. MiR-505 was found to be down-regulated in all CC cell lines. As shown in Figure 1B (all *P*<0.05), miR-505 was expressed at the lowest level in HeLa and SiHa cells, so these cell lines were selected for subsequent studies.

### Overexpression of miR-505-5p inhibits proliferation, migration, and invasion in CC cells

To evaluate the effect of miR-505-5p on CC cell proliferation, migration, and invasion, HeLa and SiHa cells were transfected with miR-505 mimics, and miR-505-5p overexpression was confirmed by qRT–PCR (*P*<0.01; Figure 2A).

**Figure 2:** MiR-505-5p expression affects migration, invasion, proliferation, and EMT process in CC cells **(A)** QRT-PCR applied to measure the relative level of miR-505-5p expression in CC cell lines (HeLa and SiHa) after transfection with miR-505 mimics, NC mimics, or control vector (^**^P<0.01; by Student’s *t*-test vs control). **(B)** The results of the CCK-8 assay performed in the control group and groups of HeLa **(C)** or SiHa cells transfected with miR-505 mimics or NC mimics are shown (^*^P<0.05, ^**^P<0.01; by ANOVA vs control). **(D)** Wound-healing assay revealed that miR-505-5p up-regulation inhibits the migration ability of HeLa **(E)** and SiHa cells. Representative images were obtained at 40× magnification at the indicated hours (^*^P<0.05, **P<0.01; by Student’s *t*-test vs control). **(F)** The effect of miR-505-5p overexpression on cell invasion, as determined by Transwell assay, obtained at 100× magnification in HeLa **(G)** and SiHa cells (^*^P<0.05, ^**^P<0.01; by Student’s *t*-test vs control). **(H)** Western blot analysis of E-cadherin, N-cadherin, and Vimentin expression following transfection with miR-505 mimics, NC mimics, or control group in HeLa **(I)** and SiHa cells. β-actin was used as an internal control (^*^P<0.05, ^**^P<0.01; by Student’s *t*-test vs control).

The effect of miR-505-5p up-regulation on CC cell proliferation was measured by CCK-8 assay. As shown in Figure 2B,C (all *P*<0.05), miR-505-5p overexpression decreased cell growth rate in both HeLa and SiHa cells, compared with control groups. The migration activity was measured by scratch wound assay. The differences in cell migration were observed at 48-h post-scratch in cells transfected with miR-505-5p, NC mimics, and those in the control group. As shown in Figure 2D,E (all *P*<0.05), miR-505-5p overexpression inhibited cell migration of HeLa and SiHa cells. Transwell assay was performed to investigate whether miR-505-5p affects the invasion ability of cancer cells. Results demonstrated that overexpression of miR-505-5p significantly reduced the invasion capacity of CC cells (all *P*<0.05; Figure 2F,G). Taken together, these data demonstrate the important role played by miR-505-5p in regulating the proliferation, migration, and invasion of CC cells *in vitro*.

### Overexpression of miR-505-5p suppresses EMT in CC cells

EMT is a vital pathologic mechanism in cancer progression. EMT markers (E-cadherin, N-cadherin, and Vimentin) were analyzed in CC cells following the overexpression of miR-505-5p. Western blot analysis demonstrated that enhanced miR-505-5p expression significantly promoted the expression of E-cadherin protein and decreased the expression of N-cadherin and Vimentin proteins (all *P*<0.05; Figure 2H,I). Consistent with this result, miR-505-5p could inhibit the EMT process and might serve as a key regulator in CC progression.

### CDK5 is up-regulated in human CC tissue samples and negatively correlates with miR-505-5p

Potential target genes of miR-505-5p were screened using a bioinformatics approach, and the 3′-UTR region of CDK5 mRNA was predicted to contain miR-505-5p complementary binding sites (Figure 3A). CDK5 was previously reported as contributing in prostate, pancreatic, lung, thyroid, and colorectal and breast cancer, as well as hepatocellular carcinoma, myeloma, and glioma [24–32]. Knockdown of CDK5 protein was found to produce increased sensitivity to cisplatin in CC treatment [33]. We suggest that CDK5 could also be implicated in CC progression.

**Figure 3:** CDK5 acts as a direct target of miR-505-5p in CC **(A)** MiR-505-5p putative binding sequence in the 3′-UTR of CDK5. **(B)** QRT-PCR was used to compare CDK5 expression levels between CC tissues and non-cancerous cervical tissues (^*^P<0.05, by Student’s *t*-test vs normal cervical tissues). **(С)** The expression levels of miR-505-5p and CDK5 were determined by qRT-PCR. The Spearman’s order correlation between miR-505-5p expression and CDK5 expression in 120 CC samples is shown (*r* = −0.300, *P*=0.025, by Pearson correlation test). **(D)** Luciferase reporter assays verified that miR-505-5p overexpression decreased the luciferase activity of cells carrying the wild-type but did not affect the mutant type 3′-UTR of CDK5 in CC cells. Relative luciferase activity was determined in HeLa and SiHa cells (^*^P<0.05, ^**^P<0.01; by Student’s *t*-test vs control). **(E)** The expression of CDK5 protein after transfection with miR-505 mimics, NC mimics, or control vector, measured by Western blot analysis in HeLa **(F)** and SiHa cell lines. β-actin was used as an internal control (^*^P<0.05; by Student’s *t*-test vs control). **(G)** Western blot assay showed CDK5 expression level in HeLa and SiHa cells after transfection with pcDNA 3.1-CDK5, pcDNA 3.1, or in control group. β-actin was used as an internal control (^*^P<0.05, ^**^P<0.01; by Student’s *t*-test vs control).

Relative CDK5 expression was determined in 120 cervical samples by qRT-PCR assays. The result showed that CDK5 was significantly up-regulated in CC samples compared with control (or histologically normal) cervical tissues (*P*<0.05; Figure 3B). The person’s order correlation was used to discover the association between miR-505-5p expression and CDK5 expression in CC samples. We determined that miR-505-5p expression was negatively correlated with the expression of CDK5 (Figure 3C). These results demonstrated that miR-505-5p-mediated oncosupressive role in CC is partly implemented through suppressing of CDK5.

### MiR-505-5p directly targets the 3′-UTR of CDK5

Luciferase reporter assays were conducted to verify that CDK5 binds to miR-505-5p directly. CDK5-WT or CDK5-MUT were co-transfected with miR-505-5p mimics, or NC mimics, in HeLa and SiHa cells. In those cells transfected with miR-505-5p, luciferase activity of CDK5-WT was significantly lower than it was for those cells within the control group (all *P*<0.05), this indicates that overexpression of miR-505-5p promoted miR-505-5p binding to its target gene CDK5 3′-UTR, so that luciferase activity was decreased. In contrast, no effect on the luciferase activity of CDK5-MUT was observed (Figure 3D). Collectively, our data reveal that miR-505-5p could combine with the specific CDK5 mRNA 3′-UTR binding sites and suppress the expression of the CDK5 gene.

### MiR-505-5p negatively regulates CDK5 protein expression in CC cells

Since CDK5 was found to be a direct target of miR-505-5p in CC cells, further experiments were performed to confirm the interaction of miR-505 with CDK5. CDK5 protein levels were evaluated in miR-505-5p mimics, NC mimics, and the control groups using Western blot analysis in HeLa and SiHa cells. Results showed that overexpression of miR-505-5p notably suppressed the protein level of CDK5; no significant effect was found in NC mimics or the control groups (all *P*<0.05; Figure 3E,F). These findings indicated that miR-505-5p down-regulates the expression of CDK5 gene by directly targeting CDK5 3′-UTR in CC cells.

### CDK5 affects proliferation, migration, and invasion, and regulates EMT in CC cells

To determine the role of CDK5 in the regulation of CC cell invasion, migration, proliferation, and EMT, HeLa and SiHa cells were transfected with pcDNA 3.1-CDK5 or with empty vector. Western blot demonstrated the efficiency of CDK5 overexpression (all *P*<0.05; Figure 3G).

CCK-8 proliferation assays were performed to detect cell viability, and we observed enhanced cell viability in pcDNA3.1-CDK5 transfected cells (all *P*<0.05; Figure 4A,B). To assess the effects of CDK5 on cell migration and invasion, scratch wound and transwell assays were performed. The cells transfected with pcDNA 3.1-CDK5 showed increased migratory and invasive abilities, compared with the cells transfected with empty vector (all *P*<0.05; Figure 4C–F). Further we studied whether CDK5 influenced EMT in CC cells. Western blot analysis demonstrated that in the group transfected with pcDNA 3.1-CDK5, both HeLa and SiHa cells exhibited a significantly decreased level of E-cadherin, a cell–cell adhesion protein, while N-cadherin and Vimentin were increased (all *P*<0.05; Figure 4G,H).

**Figure 4:** CDK5 expression affects migration, invasion, proliferation, and EMT process in CC cells **(A)** CCK-8 assay demonstrated that CDK5 transfection enhanced cell proliferation in both Hela **(B)** and SiHa cell lines (^*^P<0.05, ^**^P<0.01; by ANOVA vs control). **(C)** Wound-healing assay showed that CDK5 overexpression increases the migration ability of HeLa **(D)** and SiHa cells. Representative images were obtained at 40× magnification at the indicated hours (^*^P<0.05, ^**^P<0.01; by Student’s *t*-test vs control). **(E)** The effect of CDK5 overexpression on cell invasion, as determined by Transwell assay, obtained at 100× magnification in HeLa **(F)** and SiHa cells (^*^P<0.05, ^**^P<0.01; by Student’s *t*-test vs control). **(G)** Western blot analysis of E-cadherin, N-cadherin, and Vimentin expression in HeLa **(H)** and SiHa cells after transfection with pcDNA 3.1-CDK5, pcDNA 3.1, or in control group. β-actin was used as an internal control (^*^P<0.05, ^**^P<0.01; by Student’s *t*-test vs control).

### MiR-505-5p inhibits proliferation, migration, invasion, and EMT in CC cells by targeting CDK5

To investigate whether miR-505-5p suppresses CC cell invasion, migration, proliferation, and EMT through binding to CDK5, miR-505 mimic/NC mimics and pcDNA3.1-CDK5 (generated for CDK5 overexpression)/pcDNA 3.1 were co-transfected into HeLa and SiHa cells.

Further, CCK-8, scratch-wound and transwell assays were conducted. Cell proliferation, migration, and invasion activities were highest in the control group when HeLa and SiHa cells were transfected with pcDNA 3.1 and NC mimics. MiR-505-5p overexpression caused considerably decreased cell proliferation, migration, and invasion properties; however, CDK5 was found to partially antagonize this effect (all *P*<0.05; Figure 5A–F).

**Figure 5:** CDK5 partly attenuates the effects of MiR-505-5p overexpression in CC cells **(A)** Following transfection with pcDNA 3.1-CDK5 or pcDNA 3.1, together with miR-505 mimics or NC mimics, CCK-8 assays were performed in HeLa **(B)** and SiHa cells (^*^P<0.05, by ANOVA miR-505 mimics vs control; ^*^P<0.05, by ANOVA miR-505 mimics vs miR-505 mimics+CDK5). The graph depicts the percentages of cells for each sample at 72 h following transfection. OD values measured at 490 nm. **(C)** Scratch wound assay was performed in HeLa **(D)** and SiHa cells. Representative images were obtained at 40× magnification at the indicated hours (^**^P<0.01, by Student’s *t*-test miR-505 mimics vs control; ^*^P<0.05, by Student’s *t*-test miR-505 mimics vs miR-505 mimics+CDK5; ^*^P<0.05, by Student’s *t*-test miR-505 mimics+CDK5 vs control). **(E)** Results of transwell invasion assay, obtained at 100× magnification in HeLa cells (^**^P<0.01, by Student’s *t*-test miR-505 mimics vs control; ^*^P<0.05, by Student’s *t*-test miR-505 mimics+CDK5 vs control; ^**^P<0.01, by Student’s *t*-test miR-505 mimics vs miR-505 mimics+CDK5). **(F)** Results of transwell invasion assay, obtained at 100× magnification in SiHa cells (^**^P<0.01, by Student’s *t*-test miR-505 mimics vs control; ^*^P<0.05, by Student’s *t*-test miR-505 mimics vs miR-505 mimics+CDK5). **(G)** Western blot analysis of E-cadherin, N-cadherin, and Vimentin expression in HeLa cells. β-actin was used as an internal control (^**^P<0.01, by Student’s *t*-test miR-505 mimics vs control; ^*^P<0.05, by Student’s *t*-test miR-505 mimics vs miR-505 mimics+CDK5). **(H)** Western blot analysis of E-cadherin (^**^P<0.01, by Student’s *t*-test miR-505 mimics vs control; ^*^P<0.05, by Student’s *t*-test miR-505 mimics vs miR-505 mimics+CDK5; ^**^P<0.01, by Student’s *t*-test miR-505 mimics+CDK5 vs control), N-cadherin (^**^P<0.01, by Student’s *t*-test miR-505 mimics vs control; ^*^P<0.05, by Student’s *t*-test miR-505 mimics vs miR-505 mimics+CDK5), and Vimentin (^**^P<0.01, by Student’s *t*-test miR-505 mimics vs control; ^*^P<0.05, by Student’s *t*-test miR-505 mimics vs miR-505 mimics+CDK5) expression in SiHa cells. β-actin was used as an internal control.

Subsequently, we examined the levels of EMT-related proteins by Western blot assay. Overexpression of miR-505-p in HeLa and SiHa cells significantly up-regulated E-cadherin relative expression and down-regulated N-cadherin and Vimentin expression compared with the control group (all *P*<0.05). As shown in Figure 5G,H, slightly up-regulated epithelial marker E-cadherin, and downregulated mesenchymal markers N-cadherin and Vimentin were found in pcDNA 3.1-CDK5 and miR-505 mimics group. Taken together, the aforementioned data strongly suggest that miR-505-5p inhibits HeLa and SiHa cell proliferation, migration, invasion, and EMT by down-regulating CDK5.

## Discussion

Understanding of CC development and progression mechanisms improves every year due to an increasing number of in-depth researches. However, morbidity and fatality rates remain high, with high invasion and metastasis of CC tumors being the main causes of death [34]. The functions and therapeutic potential of cancer-related miRNAs have drawn considerable attention in recent years. Currently, miRNAs are considered as an important family of molecules with promising perspectives for cancer therapy. The ability of miRNA to modulate expression and activity *in vivo*, through miRNA mimics or antimiRs, provides an opportunity for the development of innovative therapeutic approaches. Accumulating evidence has demonstrated that miRNAs play a crucial role in various physiological processes, including invasion, metastasis, the regulation of cell growth, and drug resistance [35,36]. Accordingly, miRNAs might be used for cancer diagnosis, personalized treatments, and estimations of disease prognoses. A comprehensive understanding of the mechanisms of miRNA in CC is crucial.

Many miRs have been discovered in CC. Chen et al. [37] determined the expression levels of 1450 microRNAs in CC and normal cervical tissues. Hybridization array result showed that 89 microRNAs were differentially expressed, among them 62 were up-regulated and 27 down-regulated. Furthermore, serum microRNAs miR-1246, miR-20a, miR-2392, miR-3147, miR-3162-5p, and miR-4484 were reported as predicting lymph node metastasis in patients with CC. A meta-analysis undertaken by Li et al. [38] described 195 up-regulated miRNAs and 96 microRNAs that were down-regulated in CC tissues when compared with normal cervical specimens. Numerous recent studies have demonstrated that miRNA level in CC tissues could serve as a potential tumor biomarker. For instance, a low miR-1254 level has been associated with significantly poorer overall survival and recurrence-free survival of patients with CC [39]. Furthermore, MiR-200c has been found to be down-regulated in cervical carcinoma tissues and cell lines, and its overexpression suppressed CC cell growth and metastasis by targeting MAP4K4 [40]. MiR-143 was decreased in CC cells and tissues, and inhibited cell invasion and migration by targeting GOLM1 [41]. MiR-214 acts as a tumor suppressor targeting EZH2 in CC, while low expression of miR-214 is positively associated with tumor stage and differentiation [42]. In the short time since the discovery of miRNAs, therapeutic approaches to modulate their activity and expression level through miRNA mimics or anti-miRs have undergone considerable development, with some successful phase I trials and ongoing phase II trials [36]. Results from preclinical studies suggest that miRs might be used as cancer diagnostic markers and as anticancer therapy against CC.

Increasing evidence indicates that aberrant expression of miR-505-5p plays a significant role in carcinogenesis. A previous study showed that the down-regulation of miR-505-5p in breast tumors tissues was one of the most valuable non-invasive biomarkers for distinguishing patients with breast cancer at an early stage [17]. Another study has demonstrated that miR-505-5p regulates migration, invasion, and *in vivo* metastasis formation in colorectal cancer by targeting S100 calcium-binding protein A4 [15]. Piwecka et al. [11] found that miR-505-5p is dysregulated in malignant glioma tissues.

In the present study, we detected the expression of miR-505-5p in patients’ CC and healthy tissues and found that the expression of miR-505-5p was significantly decreased in CC samples. The present study also revealed a correlation between miR-505-5p expression level and clinicopathological characteristics of patients with CC. Through statistical analysis, a strong connection between miR-505-5p expression and FIGO stage, tumor size, lymph node metastasis, and histology grade was discovered in patients with CC.

Furthermore, overexpression of miR-505-5p significantly inhibited cell proliferation, migration, invasion, and EMT *in vitro*. Taken together, these data indicate that miR-505-5p functions as a tumor suppressor gene and that it inhibits CC malignant progression. To investigate the molecular mechanism by which miR-505-5p regulates CC progression, we found binding sites between miR-505-5p and CDK5, subsequently carrying out a follow-up study using bioinformatics analysis. In summary, by binding to the 3′-UTR of CDK5, miR-505-5p could suppress proliferation, migration, invasion, and EMT of CC cells.

CDK5 is a protein kinase involved in the development and progression of human cancers by regulating cell transformation, proliferation, invasion, and migration. CDK5 activity has also been reported as being implicated in metastasis, angiogenesis, and apoptosis [25,29,30]. Expression of CDK5 is increased in most types of human malignancies when compared with its expression in healthy tissues [31]. Previous studies have confirmed that CDK5 regulates tumorigenicity and systemic metastasis in prostate, pancreas, colorectal, and breast cancer, as well as in glioma. Moreover, it is suggested that CDK5 protein serves as a universal tumor biomarker for identifying patients with poor clinical outcomes [28,32]. CDK5 loss leads to increased drug sensitivity and may allow the identification of patients’ responding to antitumor treatment [29,31]. CDK5 activity has also been found to mediate cell migration and invasion in prostate, lung, and thyroid cancer [24,26,27]; this is consistent with the findings of our study.

Taken together, our results demonstrate a new regulatory mechanism of CDK5 targeting by miR-505-5p. These findings suggest miR-505-5p as a potential molecular marker for the diagnosis and target treatment of CC, and enhance the current understanding of the role played by miR-505-5p in CC.

## Conclusion

This is, to our knowledge, the first study that has focused on investigating a mechanism of miR-505-5p functioning in CC. We identified CDK5 as a target of miR-505-5p, exploring its functional impact on proliferation, invasion, migration, and EMT *in vitro*.

Our results may provide a basis for further research into miR-505-5p potential in CC and could be used for improving diagnostic and therapeutic approaches to this disease.

## Availability of data and materials

All data generated or analyzed during the present study are included in this published article.

## Abbreviations

CC: cervical cancer
CCk-8: cell counting kit-8
CDK5: cyclin-dependent Kinase 5
CDK5-WT: wild-type CDK5
DMEM: Dulbecco’s Modified Eagle’s Medium
FBS: phosphate-buffered saline
FIGO: International Federation of Gynecology and Obstetrics
miR: microRNA
miR-505: microRNA-505
NC: negative control
OD: optical density
PBS: phosphate-buffered saline
qRT-PCR: quantitative real-time polymerase chain PCR
S.D.: standard deviation
TBST: Tris-buffered saline, 0.1% Tween 20
UTR: untranslated region
